The article "A Hybrid Method to Predict Postoperative Survival of Lung Cancer Using Improved SMOTE and Adaptive SVM" was published in 2021. Journal: Comput Math Methods Med.

# A Hybrid Method to Predict Postoperative Survival of Lung Cancer Using Improved SMOTE and Adaptive SVM

**DOI:** 10.1155/2021/2213194

**Published:** 2021-09-10

**Authors:** Jiang Shen, Jiachao Wu, Man Xu, Dan Gan, Bang An, Fusheng Liu

**Affiliations:** ^1^College of Management and Economics, Tianjin University, Tianjin 300072, China; ^2^Business School, Nankai University, Tianjin 300071, China; ^3^School of Economics and Management, Hebei University of Technology, Tianjin 300071, China

## Abstract

Predicting postoperative survival of lung cancer patients (LCPs) is an important problem of medical decision-making. However, the imbalanced distribution of patient survival in the dataset increases the difficulty of prediction. Although the synthetic minority oversampling technique (SMOTE) can be used to deal with imbalanced data, it cannot identify data noise. On the other hand, many studies use a support vector machine (SVM) combined with resampling technology to deal with imbalanced data. However, most studies require manual setting of SVM parameters, which makes it difficult to obtain the best performance. In this paper, a hybrid improved SMOTE and adaptive SVM method is proposed for imbalance data to predict the postoperative survival of LCPs. The proposed method is divided into two stages: in the first stage, the cross-validated committees filter (CVCF) is used to remove noise samples to improve the performance of SMOTE. In the second stage, we propose an adaptive SVM, which uses fuzzy self-tuning particle swarm optimization (FPSO) to optimize the parameters of SVM. Compared with other advanced algorithms, our proposed method obtains the best performance with 95.11% accuracy, 95.10% *G*-mean, 95.02% F1, and 95.10% area under the curve (AUC) for predicting postoperative survival of LCPs.

## 1. Introduction

Lung cancer (LC) is the deadliest cancer in the world. More than 85% of lung cancer patients are diagnosed with non-small-cell LC [1]. Surgical resection is the standard and most effective treatment for LC stage I, stage II, and nonsmall cell stage III A [1]. A major problem of the clinical decision on LC operation is to select candidates for surgery based on the patient's short-term and long-term risks and benefits, where survival time is one of the most important measures. Accurately predicting a patient's survival after surgery can help doctors make better treatment decisions. At the same time, it can help patients better understand their conditions to have good psychological expectations and financial preparation.

In recent years, more and more data-driven methods have been used to predict the postoperative survival of LCPs. In terms of statistical methods, Kaplan–Meier curves, multivariable logistic regression, and Cox regression are the three most widely used statistical methods to predict survival or complications for LCPs [2]. However, taking into account the shortcomings of traditional statistical methods and the incompleteness of medical data, data mining and machine learning techniques are introduced in recent years. Mangat and Vig [3] proposed an association rule algorithm based on a dynamic particle swarm optimizer, and the classification accuracy is 82.18%. Saber Iraji [4] compared the accuracy of adaptive fuzzy neural networks, extreme learning machine, and neural networks for predicting the 1-year postoperative survival of LCPs. The results show that sensitivity (90.05%) and specificity (81.57%) of an extreme learning machine are the highest, respectively. Tomczak et al. [5] used the boosted support vector machine (SVM) algorithm to predict the postoperative survival of LCPs. This algorithm combines the advantages of ensemble learning and cost-sensitive SVM, and the *G*-mean can reach 65.73%. As can be seen from the previous research, most of them ignore the impact of imbalanced data distribution, which may reduce the performance of classifiers.

The article "A Hybrid Method to Predict Postoperative Survival of Lung Cancer Using Improved SMOTE and Adaptive SVM" was published in 2021. Journal: Comput Math Methods Med.

Class imbalance refers to the phenomenon in which one class of data in a dataset is much larger than the others [6]. Standard machine learning classifiers are effective for balanced data, but they are not good for imbalanced data. Specifically, with the progress of medical technology, the number of long-term survivors after surgery for LCPs is much larger than that of short-term deaths. This will lead to higher prediction accuracy for survivors (majority class) and poorer recognition for deceases (minority class). Therefore, it is necessary to propose a method that has good classification performance for both survivors and deceased ones for predicting postoperative survival of LCPs.

During the past decades, the imbalanced data classification problem has widely become a matter of concern and has been intensively researched. The existing papers on imbalanced data processing methods have two main research directions: data level and algorithm level [7]. The data-level processing methods create a balanced class distribution by resampling the input data. Algorithm-level processing methods mainly involve two aspects: ensemble learning and cost-sensitive learning. Among these imbalanced data processing methods, the synthetic minority oversampling technique (SMOTE) is one of the most widely used methods, as it is relatively simple and effective [8]. However, it is likely to be unsatisfactory or even counterproductive if SMOTE is used alone, which is because its blind oversampling ignores the distribution of samples, such as the existence of noise [9, 10]. To solve this problem, many approaches are proposed to improve SMOTE. Ramentol et al. [11] combined rough set theory with SMOTE and proposed the SMOTE-RSB algorithm. SMOTE-RSB first uses SMOTE for oversampling and then removes noise and outliers in the dataset based on rough set theory. SSMNFOS [12] is a hybrid method based on stochastic sensitivity measurement (SSM) noise filtering and oversampling, which can improve the robustness of the oversampling method with respect to noise samples. The CURE-SMOTE [13] uses CURE (clustering using representatives) to cluster minority samples for removing noise and outliers and then uses SMOTE to insert artificial synthetic samples between representative samples and central samples to balance the dataset. However, most of these methods need to set the noise threshold through prior parameters, which increases the risk of misidentification of noise. In addition, some researchers consider ensemble filtering methods, which have been proven to be generally more efficient than single filters [14]. In this paper, we propose to use the cross-validated committees filter (CVCF) to detect and remove noise before applying SMOTE and record this method as CVCF-SMOTE. CVCF is an ensemble-based filter, which can reduce the risk of error in the threshold setting of prior parameters [15].

The article "A Hybrid Method to Predict Postoperative Survival of Lung Cancer Using Improved SMOTE and Adaptive SVM" was published in 2021. Journal: Comput Math Methods Med.

In addition, SVM as one of the most advanced classifiers has not been well used to predict postoperative survival of LC. In the previous research, SVM has been widely used in statistical classification and regression analysis due to its excellent performance [16]. Considering the limitations of SVM on imbalanced data, some studies combine resampling technology and SVM to deal with imbalanced data. D'Addabbo and Maglietta [17] proposed a method combining parallel selective sampling and SVM (PSS-SVM) to process imbalanced big data. Experimental results show that the performance of PSS-SVM is better than that of SVM and RUSBoost classifiers. Huang et al. [18] designed an undersampling technique based on clustering and combined it with optimized SVM to deal with imbalanced data. The classification performance of SVM is improved by the linear combination of SVM based on a mixed kernel. Fan et al. [19] proposed a hybrid technology combining principal component analysis (PCA), SMOTE, and SVM to diagnose chiller fault. Experimental results prove that this hybrid technology can improve the overall performance of chiller fault diagnosis.

However, these studies usually require a manual setting of SVM parameters, which may lead to failure to obtain the best experimental results. The standard SVM has a limitation that its performance depends on the selection of initial parameters. Some studies optimize the parameters of SVM through evolutionary calculations which have achieved good results. In these optimization algorithms, the particle swarm optimization- (PSO-) optimized SVM has been widely used with promising results due to its simplicity and fast convergence [20]. With the development of PSO technology, some improved PSO algorithms are used to optimize SVM. Wei et al. [21] proposed a binary PSO-optimized SVM method for feature selection, which overcomes the problem of premature convergence and obtained high-quality features. A switching delayed particle swarm optimization- (SDPSO-) optimized SVM is proposed to diagnose Alzheimer's disease [22]. Experimental results show that the proposed method outperforms several other variants of SVM and has obtained excellent classification accuracy. However, these methods often require parameter settings for PSO or improved PSO, such as particle size and inertial weight. In general, getting the best settings is complicated and time-consuming. If the PSO parameters are set improperly, it will even reduce the performance of the SVM.

The article "A Hybrid Method to Predict Postoperative Survival of Lung Cancer Using Improved SMOTE and Adaptive SVM" was published in 2021. Journal: Comput Math Methods Med.

In recent years, many new metaheuristics techniques have been proposed, such as Monarch Butterfly Optimization (MBO) [23], slime mould algorithm [24], Moth Search (MS) [25], Hunger Games Search (HGS) [26], and Harris Hawks Optimizer (HHO) [27]. However, most of these methods require users to tune parameters to achieve satisfactory performance. Fuzzy self-tuning PSO (FPSO) is a kind of setting-free adaptive PSO proposed in recent years [28]. The advantage of FPSO is that every particle is adaptively adjusted during the optimization process without any PSO expertise and parameter settings. Moreover, experimental results show that FPSO is better than several previous competitors in convergence speed and finding optimal solution aspects. Based on the above considerations, the FPSO algorithm is exploited to optimize the parameters of SVM, which leads to a novel FPSO-SVM classification algorithm.

Based on the improved SMOTE and FPSO-SVM, we propose a two-stage hybrid method to improve the performance of the postoperative survival prediction of LCPs. In the first stage, CVCF is used to remove noise samples to improve the performance of SMOTE. Then, SMOTE is adopted to handle the imbalanced nature of the dataset. In the second stage, we apply FPSO-SVM to predict the postoperative survival of LCPs. The experimental results show that the proposed hybrid method outperforms other comparative state-of-the-art algorithms. This hybrid method can effectively improve the accuracy of survival prediction after LC surgery and provide reliable medical decision-making support for doctors and patients. Our contributions are summarized as follows:

- A novel hybrid method that combines improved SMOTE with adaptive SVM is proposed for predicting postoperative survival of LCPs
- We apply CVCF to clean up data noise to improve the performance of SMOTE
- FPSO is used to optimize the parameters of SVM and achieve an adaptive SVM
- The proposed hybrid method not only performs higher predictive accuracy than other compared algorithms for predicting postoperative survival of LCPs but also has better *G*-mean, F1, and area under the curve (AUC)

The rest of this paper is as follows: Section 2 shows the materials and methods. The experiment design, performance metrics, and experimental results are described in Section 3. A brief summary is described in Section 4.

The article "A Hybrid Method to Predict Postoperative Survival of Lung Cancer Using Improved SMOTE and Adaptive SVM" was published in 2021. Journal: Comput Math Methods Med.

## 2. Materials and Methods

### 2.1. Data Description

In this paper, the thoracic surgery dataset in Zięba et al. [5], is selected to predict the postoperative survival of LCPs. Data were collected from the Wroclaw Thoracic Surgery Center. These patients underwent lung resection for primary LC from 2007 to 2011. It contains 470 samples with an imbalance rate of 5.71. There are 400 patients who survived more than one year and 70 patients who survived less than one year in this dataset.  Table 1 shows the features of the dataset. These features were selected from 36 preoperative predictors by the information gain method and were used to predict the postoperative survival expectancy. Our task is to predict whether the survival time in patients after surgery was greater than one year.

### 2.2. Data Preprocessing

#### 2.2.1. CVCF for Noise Cleaning

Although SMOTE is one of the most widely used methods for imbalanced data processing, it has some drawbacks in dealing with data noise. A major concern is that SMOTE may exacerbate the presence of noise in the data, as shown in Figure 1. Given the good performance of CVCF, we consider using it to improve SMOTE.

The CVCF algorithm is a well-known representative of an ensemble-based noise filter [29]. It induces multiple single classifiers by means of cross-validation. Afterward, samples mislabeled by all classifiers (or most classifiers) will be marked as noise and removed from the dataset. Choosing an appropriate base classifier is a key operation to ensure the excellent performance of CVCF. In this paper, we choose the C4.5 algorithm as the base classifier of CVCF because it has better robustness to noise data and suitability for ensemble learning [30, 31].

C4.5 is an improved version of the ID3 algorithm [32]. It improves ID3 by handing numeric attributes and missing values and by introducing pruning. In addition, essentially different from the ID3, the information gain ratio is used to select split attributes in C4.5, which can be denoted by

(1) $$\begin{array}{c} \text{InfoGainRatio}\left(S,A\right)=\frac{\text{InfoGain}\left(S,A\right)}{\text{SpiltInfo}\left(S,A\right)}, \end{array}$$

where InfoGainRatio(*S*, *A*) represents the information gain ratio of attribute *A* in dataset *S*. InfoGain(*S*, *A*) is the information gain of dataset *S* after splitting through attribute *A* and can be denoted by

(2) $$\begin{array}{c} \text{InfoGain}\left(S,A\right)=\text{Info}\left(S\right)-\text{Info}\left(S,A\right), \end{array}$$

where Info(*S*) is the entropy of dataset *S*. Info(*S*, *A*) is the conditional entropy about attribute *A*. SpiltInfo(*S*, *A*) denotes the splitting information of attribute *A* and is expressed by

(3) $$\begin{array}{c} \text{SpiltInfo}\left(S,A\right)=-\overset{m}{\underset{i=1}{\sum }}\frac{\left|S_{i}\right|}{\left|S\right|}\log_{2}\frac{\left|S_{i}\right|}{\left|S\right|}, \end{array}$$

where |*S*| represents the number of samples of dataset *S*. |*S*_*i*_| indicates the number of samples of subset *i* after the original dataset is divided into *m* subsets according to the attribute value of *A*.

The article "A Hybrid Method to Predict Postoperative Survival of Lung Cancer Using Improved SMOTE and Adaptive SVM" was published in 2021. Journal: Comput Math Methods Med.

#### 2.2.2. SMOTE to Balance Data

The core idea of SMOTE is to insert artificial samples of similar values into the minority class, thereby improving the imbalanced distribution of classes. More specifically, the sampling ratio is set firstly, and then, the *k* nearest neighbors of each minority sample are found. Finally, according to equation (4), one of the neighbors is randomly selected to generate a synthetic sample that is put back into the dataset until the sampling number reaches the set ratio. The synthesized new sample is calculated as follows:

(4) $$\begin{array}{c} X_{new}=X+\partial \left(X_{i}‐X\right),\;\partial \in \left(0,1\right), \end{array}$$

where **X**_**new**_ represents a new synthetic sample, **X** is the feature vector for each sample in the minority class, and **X**_**i**_ is the *i*-th nearest neighbor of sample **X**. *∂* is a random number between 0 and 1.

### 2.3. The Proposed FPSO-Optimized SVM (FPSO-SVM)

#### 2.3.1. SVM

SVM is a supervised learning classifier based on statistical theory and structural risk optimization [33]. SVM is not prone to overfitting and can handle high-dimensional data well. The principle of SVM is to map the original data to a high-dimensional space to discover a hyperplane that maximizes the margin determined by the support vectors. Suppose there is a dataset *D* = {(**x**_1_, *y*_1_), (**x**_2_, *y*_2_), ⋯, (**x**_**n**_, *y*_*n*_)}. The optimal hyperplane of dataset *D* can be expressed as

(5) $$\begin{array}{c} a^{T}x+b=0, \end{array}$$

where **a**^*T*^ is the weight vector and *b* represents the bias.

The article "A Hybrid Method to Predict Postoperative Survival of Lung Cancer Using Improved SMOTE and Adaptive SVM" was published in 2021. Journal: Comput Math Methods Med.

For nonlinear problems, the above-mentioned optimal hyperplane can be transformed into

(6) $$\begin{array}{c} \left\{\begin{array}{c} \underset{a,b}{\min}\\ \text{s}.\text{t}. \end{array}\right.\begin{array}{c} \frac{1}{2}a^{T}a‐C\overset{n}{\underset{i=1}{\sum }}\zeta_{i},\\ y_{i}\left(a^{T}\cdot x_{i}+b\right)\geq 1-\zeta_{i},\;\zeta_{i}\geq 0\;i=1,2,\cdots ,n, \end{array} \end{array}$$

where *C* is the penalty factor and *ζ*_*i*_ is the slack variable. The above constrained objective function can satisfy the KKT condition by introducing the Lagrange formulation. The original objective function is transformed into

(7) $$\begin{array}{c} \left\{\begin{array}{c} \min\frac{1}{2}\overset{n}{\underset{i=1}{\sum }}\overset{n}{\underset{j=1}{\sum }}y_{i}y_{j}\beta_{i}\beta_{j}\left(x_{i}\cdot x_{j}\right)-\overset{n}{\underset{i=1}{\sum }}\beta_{i},\\ \text{s}.\text{t}.\;\overset{n}{\underset{i=1}{\sum }}\beta_{i}y_{i}=0,\;0\leq \beta_{i}\leq C,\;i,j=1,2,\cdots ,n, \end{array}\right. \end{array}$$

where *β* is a Lagrangian multiplier. According to the previous experimental experience, a larger value of *C* means a larger separation interval and a greater generalization risk. Conversely, when the value of *C* is too small, it is easy to have an underfitting problem.

Finally, the decision function is shown in

(8) $$\begin{array}{c} f\left(x\right)=\mathrm{sgn}\left(\overset{n}{\underset{i=1}{\sum }}\beta_{i}^{*}y_{i}K<x_{i}\cdot x_{j}>+b^{*}\right), \end{array}$$

where *β*_*i*_^∗^ and *b*^∗^ are the optimal Lagrangian multiplier and optimal value of *b*, respectively, and sgn(·) represents a symbolic function. *K* < **x**_*i*_ · **x**_*j*_> is a kernel function. Usually, the radial basis function (RBF) kernel function is selected for SVM, which can be expressed as

(9) $$\begin{array}{c} K<x_{i}\cdot x_{j}>=\exp\left(-\gamma {\left\|x_{i}-x_{j}\right\|}^{2}\right), \end{array}$$

where *γ* is the kernel parameter. The classification performance of SVM depends heavily on the setting of penalty factor *C* and kernel parameter *γ*. Therefore, parameter setting is a key step in applying SVM.

#### 2.3.2. FPSO-SVM Model

In order to make SVM have better classification performance, we use FPSO to optimize the penalty factor *C* and kernel parameter *γ* of SVM, called FPSO-SVM. The classification accuracy is taken as the fitness function of FPSO, which is defined as

(10) $$\begin{array}{c} \text{Fitness}=\text{Accuracy}=\frac{\text{TP}+\text{TN}}{\text{TP}+\text{TN}+\text{FP}+\text{FN}}, \end{array}$$

where TP, TN, FP, and FN represent four different classification results which are shown in Table 2.

The article "A Hybrid Method to Predict Postoperative Survival of Lung Cancer Using Improved SMOTE and Adaptive SVM" was published in 2021. Journal: Comput Math Methods Med.

FPSO is a fully adaptive version of PSO, which calculates the inertia weight, learning factor, and velocity independently for each particle based on fuzzy logic. The outstanding advantages of FPSO are that it does not require any prior knowledge about PSO and its optimization performance and convergence speed are better than those of PSO.

In FPSO, first, the number of particle swarms is set to $N=10+2\sqrt{M}$ based on the heuristic [34, 35]. Here, *M* is the dimension of the optimization problem. In this paper, since there are two SVM parameters that need to be optimized, *M* = 2 and *N* = 12 (round down). After initializing the particles, we need to update them according to the position and velocity of the particles. Let **x**_*i*_^*k*^ and **v**_*i*_^*k*^ be the velocity and position of the *i*-th particle at the *k*-th iteration, respectively. At the (*k* + 1)-th iteration, the velocity **v**_*i*_^*k*+1^ and position **x**_*i*_^*k*+1^ of the *i*-th particle can be defined as

(11) $$\begin{array}{c} v_{i}^{k+1}=w_{i}^{k}\cdot v_{i}^{k}+c_{{\text{soc}}_{i}}^{k}\cdot r_{1}\cdot \left(x_{i}^{k}-g^{k}\right)+c_{{\text{cog}}_{i}}^{k}\cdot r_{2}\cdot \left(x_{i}^{k}‐b_{i}^{k}\right),\;i=1,2\cdots ,12, \end{array}$$

(12) $$\begin{array}{c} x_{i}^{k+1}=x_{i}^{k}+v_{i}^{k+1}, \end{array}$$

where *w*_*i*_^*k*^ is the inertia weight of particle *i* at the *k*-th iteration and *c*_soc_*i*__^*k*^ and *c*_cog_*i*__^*k*^ are social and cognitive factors of particle *i* at the *k*-th iteration, respectively. In FPSO, unlike conventional PSO, the values of *w*_*i*_^*k*^, *c*_soc_*i*__^*k*^, and *c*_cog_*i*__^*k*^ are not fixed but are calculated separately for different particles at each iteration. **r**_1_ and **r**_2_ are two random vectors, respectively. **b**_*i*_^*k*^ and **g**^*k*^ are the position of the *i*-th particle and the best global position in the swarm at the *k*-th iteration.

The maximum velocity (*v*_max_*m*__) and minimum velocity (*v*_min_*m*__) of all particles in the *m*-th dimension are defined as

(13) $$\begin{array}{c} v_{\max_{m}}=\eta \cdot \left(b_{\max_{m}}-b_{\min_{m}}\right),\;\eta \in \left(0,1\right]. \end{array}$$

(14) $$\begin{array}{c} v_{\min_{m}}=\lambda \cdot \left(b_{\max_{m}}-b_{\min_{m}}\right),\;\lambda \in \left(0,1\right], \end{array}$$

where *b*_max_*m*__ and *b*_min_*m*__ represent upper and lower bounds of the *m*-th dimension for the optimization problem, respectively. *η* and *λ* (*η* > *λ*) are two coefficients determined by linguistic variables, in order to clamp *v*_max_*m*__ and *v*_min_*m*__ of each particle.

The article "A Hybrid Method to Predict Postoperative Survival of Lung Cancer Using Improved SMOTE and Adaptive SVM" was published in 2021. Journal: Comput Math Methods Med.

In order to get the *w*, *c*_soc_, *c*_cog_, *η*, and *λ* values of each particle in each iteration, two concepts are introduced: the distance between each particle and the global optimal particle and the fitness increment of each particle relative to the previous iteration.

The distance between any two particles in the *k*-th iteration is expressed as

(15) $$\begin{array}{c} \delta \left(x_{i}^{k},x_{j}^{k}\right)={\left\|x_{i}^{k}-x_{j}^{k}\right\|}_{2}=\sqrt{\overset{2}{\underset{m=1}{\sum }}{\left(x_{i,m}^{k}-x_{j,m}^{k}\right)}^{2}},\;i,j=1,2,\cdots ,12. \end{array}$$

The function *ϕ* represents the normalized fitness increment of particle *i* for the previous iteration, which is calculated as

(16) $$\begin{array}{c} \phi \left(x_{i}^{k+1},x_{i}^{k}\right)=\frac{\delta \left(x_{i}^{k+1},x_{i}^{k}\right)}{\delta_{\max}}\cdot \frac{\min\left\{f\left(x_{i}^{k+1}\right),f_{\text{wor}}\right\}-\min\left\{f\left(x_{i}^{k}\right),f_{\text{wor}}\right\}}{\left|f_{\text{wor}}\right|}, \end{array}$$

where *δ*_max_ is the diagonal length of the rectangle formed by the search space. *f*_wor_ is the worst fitness value.

The linguistic variable of function *δ* is defined as Same, Near, and Far, which is used to measure the distance from a particle to the global best particle. The trapezoid membership function of Same is defined as

(17) $$\begin{array}{c} \delta =\left\{\begin{array}{cc} 1, & \text{if }0\leq \delta <\delta_{1},\\ \frac{\delta_{2}-\delta }{\delta_{2}-\delta_{1}}, & \text{if }\delta_{1}\leq \delta <\delta_{2},\\ 0, & \text{if }\delta_{2}\leq \delta \leq \delta_{\max}. \end{array}\right. \end{array}$$

The triangle membership function of Near is defined as

(18) $$\begin{array}{c} \delta =\left\{\begin{array}{cc} 0, & \text{if }0\leq \delta <\delta_{1},\\ \frac{\delta -\delta_{1}}{\delta_{2}-\delta_{1}}, & \text{if }\delta_{1}\leq \delta <\delta_{2},\\ \frac{\delta_{3}-\delta }{\delta_{3}-\delta_{2}}, & \text{if }\delta_{2}\leq \delta <\delta_{3},\\ 0, & \text{if }\delta_{3}\leq \delta \leq \delta_{\max}. \end{array}\right. \end{array}$$

The trapezoid membership function of Far is defined as

(19) $$\begin{array}{c} \delta =\left\{\begin{array}{cc} 0, & \text{if }0\leq \delta <\delta_{2},\\ \frac{\delta -\delta_{2}}{\delta_{3}-\delta_{2}}, & \text{if }\delta_{2}\leq \delta <\delta_{3},\\ 1, & \text{if }\delta_{3}\leq \delta \leq \delta_{\max}, \end{array}\right. \end{array}$$

where *δ*_1_ = 0.2 · *δ*_max_, *δ*_2_ = 0.4 · *δ*_max_, and *δ*_3_ = 0.6 · *δ*_max_.

The linguistic variable of function *ϕ* is defined as Better, Same, and Worse, which is used to measure the improvement of a particle's fitness value for the previous iteration. The trapezoid membership function of Better can be obtained by

(20) $$\begin{array}{c} \phi =\left\{\begin{array}{cc} 1, & \text{if }\phi =-1,\\ -\phi , & \text{if}-1<\phi <0,\\ 0, & \text{if }0\leq \phi \leq 1. \end{array}\right. \end{array}$$

The triangle membership function of Same is expressed as follows:

(21) $$\begin{array}{c} \phi =1-\left|\phi \right|. \end{array}$$

The triangle membership function of Worse is as follows:

(22) $$\begin{array}{c} \phi =\left\{\begin{array}{cc} 0, & \text{if}-1\leq \phi <0,\\ \phi , & \text{if }0\leq \phi <1,\\ 1, & \text{if }\phi =1. \end{array}\right. \end{array}$$

According to the preset fuzzy rules, *w*, *c*_soc_, *c*_cog_, *η*, and *λ* have three levels including Low, Medium, and High [28].  Table 3 shows the defuzzification values of *w*, *c*_soc_, *c*_cog_, *η*, and *λ*, which are calculated by the Sugeno inference method [36]. It is defined as follows:

(23) $$\begin{array}{c} \text{output}=\frac{\sum_{r=1}^{R}\rho_{r}z_{r}}{\sum_{r=1}^{R}\rho_{r}},\;r=1,2\cdots R, \end{array}$$

where *R* represents the number of rules. *ρ*_*r*_ and *z*_*r*_ are the membership degree of the input variable and output value of the *r*-th rule, respectively.

The article "A Hybrid Method to Predict Postoperative Survival of Lung Cancer Using Improved SMOTE and Adaptive SVM" was published in 2021. Journal: Comput Math Methods Med.

Then, update the position of each particle based on the obtained values of *w*, *c*_soc_, *c*_cog_, *η*, and *λ*. Finally, recalculate the fitness of each particle, that is, accuracy of the SVM corresponding to each particle. Repeat the above process until the maximum number of iterations is reached and output SVM with the optimal parameters.

The time complexity of FPOS-SVM consists of two parts: FPSO and SVM. In FPSO, the velocity and position of each particle are calculated in each iteration. Therefore, the computational complexity of FPSO is determined by the number of iterations, the particle swarm size, and the dimensionality of each particle. Thus, FPSO requires *O*(*TNm*) time complexity, where *T* is the number of iterations of FPSO, *N* is the particle swarm size of FPSO, and *m* is the dimensionality of the optimization problem. For SVM, the optimal hyperplane is obtained by computing the distance between the support vector and the decision boundary. Then, the time complexity required for SVM is *O*(*dn*_sv_), where *d* is the input vector dimension and *n*_sv_ is the number of support vectors. In FPSO-SVM, the number of SVM computations depends on the particle swarm size and the number of iterations of FPSO. Therefore, the time complexity of FPSO-SVM is *O*(*TNm* + *TNdn*_sv_).

### 2.4. Specific Steps of the Proposed Hybrid Method for Predicting Postoperative Survival of LCPs

Based on improved SMOTE and FPSO-SVM, we propose a two-stage hybrid method to improve the performance of the postoperative survival prediction of LCPs. In the first stage, CVCF is used to remove noise samples to improve the performance of SMOTE. Then, apply SMOTE to balance data. In the second stage, FPSO-SVM is adopted to predict postoperative survival of LCPs.  Figure 2 shows the flowchart of the proposed hybrid method. The specific steps of the hybrid method are presented as follows:

1. Set CVCF to *n*-fold cross-validation. Then, the original dataset is divided into *n* subsets
2. Take a different subset from the *n* subsets each time as the testing set and the remaining *n* − 1 subsets as the training set. Therefore, a total of *n* different C4.5 classifiers are trained. Then, all the trained C4.5 classifiers will vote for each sample in the dataset. In this way, each sample has a real class label and *n* labels marked by C4.5
3. For each sample, determine whether all (or most) labels marked with C4.5 are different from the real one. If all (or most) of them are different from the real class label, the sample will be treated as noise and removed from the dataset. On the contrary, the sample is retained. Finally, all the retained samples make up a cleaned dataset
4. Oversample from the cleaned dataset with SMOTE until the class distribution of the dataset is balanced
5. After data preprocessing with CVCF-SMOTE, the new dataset is divided into a training set and a testing set
6. Set the search range for the penalty factor *C* and kernel parameter *γ*. Initialize particle swarm
7. Evaluate the fitness of each particle based on equation (10). Calculate the linguistic values of Inertia, Social, Cognitive, *η*, and *λ* according to equations (13)-(22)
8. Convert the language values of Inertia, Social, Cognitive, *η*, and *λ* into numerical values based on equation (23) and Table 3. Update the velocity and position of each particle based on equations (11) and (12)
9. Determine whether the maximum number of iterations has been reached. If it is reached, the optimized SVM is output. Otherwise, return to steps (7) and (8)
10. Apply the optimized SVM on the testing set

The article "A Hybrid Method to Predict Postoperative Survival of Lung Cancer Using Improved SMOTE and Adaptive SVM" was published in 2021. Journal: Comput Math Methods Med.

## 3. Experiments and Results

### 3.1. Experiment Design

To evaluate our proposed hybrid method, we compare it with several state-of-the-art algorithms including PSO-optimized SVM (PSO-SVM), SVM, *k*-nearest neighbor (KNN) [37], random forest (RF) [38], gradient boosting decision tree (GBDT) [39], and AdaBoost [40]. In addition, we consider six preprocessing approaches, including CVCF-SMOTE, Borderline-SMOTE (B-SMOTE) [41], Safe-Level-SMOTE (SL-SMOTE) [42], SMOTE-TL [43], SMOTE, and no preprocessing (marked as NONE), to explore the performance of our proposed CVCF-SMOTE method. B-SMOTE, SL-SMOTE, and SMOTE-TL are three representative SMOTE extensions, which can handle imbalanced data with noise. In addition, in order to better evaluate the effectiveness of the proposed hybrid method, we tested its performance on two other imbalanced data. The value range of penalty factor *C* and kernel parameter *γ* is set to [0, 30], and the maximum number of iterations is set to 30. All of these algorithms are programmed in the Python programming language, except for CVCF-SMOTE which is run in the KEEL software [44]. To eliminate randomness, experiments are repeated 10 times and the average performance is shown in this study.

### 3.2. Performance Metrics

In this section, we introduce the selected widely used imbalanced data classification performance metrics, including accuracy (defined by equation (10)), *G*-mean, F1, and AUC. They can be calculated according to the confusion matrix in Table 2.

(24) $$\begin{array}{c} G‐\text{mean}=\sqrt{\frac{\text{TP}}{\text{TP}+\text{FN}}\times \frac{\text{TN}}{\text{TN}+\text{FP}}}, \end{array}$$

(25) $$\begin{array}{c} \text{F}1=\frac{2*\text{precision}*\text{recall}}{\text{precision}+\text{recall}}, \end{array}$$

where precision = TP/(TP + FP) and recall = TP/(TP + FN). Precision can be regarded as a measure of the exactness of a classifier, while recall can be regarded as a measure of the completeness of a classifier.

AUC is defined as the area under the ROC curve and the coordinate axis. AUC is very suitable for the evaluation of imbalanced data classifiers because it is not sensitive to imbalanced distribution and error classification costs, and it can achieve the balance between true positive and false positive [45].

### 3.3. Result and Discussion

Tables 4–7 demonstrate the accuracy, *G*-mean, F1, and AUC values of different algorithms under different preprocessing methods for predicting postoperative survival of LCPs, respectively. The best experimental results of different preprocessing methods are marked in bold. We can see from Tables 4–7 that the proposed CVCF-SMOTE+FPSO-SVM model obtains the best performance among all methods with 95.11% accuracy, 95.10% *G*-mean, 95.02% F1, and 95.10% AUC. This shows that our proposed hybrid method can balance the classification accuracy of the minority class and the majority class while ensuring overall accuracy. That is, the proposed CVCF-SMOTE+FPSO-SVM method has a higher recognition rate for patients who survived after LC surgery for both longer than 1 year and less than 1 year.

In addition, it is easy to see from Tables 5–7 that the *G*-mean, F1, and AUC performances of different classifiers for the original dataset without preprocessing are extremely poor. However, it can be found from Table 4 that the classification accuracy of all the classifiers for the original dataset is higher than the accuracy after SMOTE preprocessing. This indicates susceptibility to imbalanced data; although the classifiers perform well in the majority class, it performs very poorly in the minority class. That is to say, these classifiers fail to balance the classification accuracy of LCPs whose survival time after surgery is longer than 1 year and less than 1 year.

The article "A Hybrid Method to Predict Postoperative Survival of Lung Cancer Using Improved SMOTE and Adaptive SVM" was published in 2021. Journal: Comput Math Methods Med.

For the performance after preprocessing with SMOTE, we found that the *G*-mean, F1, and AUC values of most classifiers (except SVM) are higher than those of the original dataset. However, as can be seen from Table 4, the accuracy of all classifiers with SMOTE is lower than that of the original dataset. This shows that although SMOTE can balance precision and recall, it leads to a decrease in accuracy. For the three SMOTE extensions SL-SMOTE, SMOTE-TL, and B-SMOTE, we find that B-SMOTE has the most competitive performance. B-SMOTE+FPSO-SVM obtained the experimental results second only to CVCF-SMOTE+FPSO-SVM.

Figure 3 shows the stacked histograms of accuracy, *G*-mean, F1, and AUC for different algorithms under different preprocessing methods. It can be seen from Figure 3 that our proposed CVCF-SMOTE+FPSO-SVM has the best performance in predicting postoperative survival of LCPs. The main reasons behind the experimental results are as follows: first, CVCF identifies and removes noise to improve the data quality so that blind oversampling can be reduced when applying SMOTE. Second, FPSO-SVM can search the optimal parameters of SVM adaptively, which improves the classification accuracy of SVM.

In order to further test the difference between CVCF-SMOTE+FPSO-SVM and other combination methods, a paired *t*-test was conducted among CVCF-SMOTE+FPSO-SVM and the best results under different preprocessing methods. A *p* value less than 0.05 is considered to be statistically significant in the experiment. From Table 8, it can be seen that CVCF-SMOTE+FPSO-SVM achieves significantly better results than the best results under different preprocessing methods in terms of the accuracy, F1, *G*-mean, and AUC at the prescribed statistical significance level of 5%.

We also compare the accuracy of our proposed model with previous studies as shown in Table 9. We can see from Table 9 that the accuracy of the CVCF-SMOTE+FPSO-SVM model is higher than that of other methods of the previous literature. Finally, we compare the ROC curves of different algorithms under different preprocessing methods, as shown in Figure 4. The greater the AUC value, the better the classifier performance. It can be seen that the AUC of our proposed CVCF-SMOTE+FPSO-SVM is the largest, which means that our proposed model is outperforming other comparison methods for predicting postoperative survival of LCPs.

The article "A Hybrid Method to Predict Postoperative Survival of Lung Cancer Using Improved SMOTE and Adaptive SVM" was published in 2021. Journal: Comput Math Methods Med.

In order to further prove that the performance of our proposed FPSO-SVM is superior to that of PSO-SVM, we draw the fitness curves of these two algorithms. Figures 5(a) and 5(b) show fitness curves of FPSO-SVM and PSO-SVM with CVCF-SMOTE preprocessing. As can be seen from (Figures 5(a) and 5(b)), we can clearly see that compared with PSO-SVM, FPSO-SVM not only has a higher fitting degree but also a faster convergence speed. This shows that our proposed FPSO-SVM algorithm can identify the optimal solution in the search space faster and more accurately than PSO-SVM.

### 3.4. Works on Other Datasets

To show the generalization ability of our proposed method, we apply CVCF-SMOTE+FPSO-SVM to the other two imbalanced datasets collected from KEEL (https://sci2s.ugr.es/keel/) [44].  Table 10 shows the details of the two selected datasets.

Tables 11 and 12 show the accuracy and AUC of different algorithms in different preprocessing methods on the Haberman dataset. It can be seen from Tables 11 and 12 that under different preprocessing methods, accuracy and AUC of CVCF-SMOTE+FPSO-SVM are higher than those of the comparison classifiers. As shown in Table 13, the results of the paired *t*-test also show that CVCF-SMOTE+FPSO-SVM is significantly better than the best experimental results under different preprocessing methods on the Haberman dataset. For the appendicitis dataset, it can be seen from Tables 14 and 15 that CVCF-SMOTE+FPSO-SVM also obtains the highest accuracy and AUC value compared to other preprocessing methods and classifier combinations. As can be seen from Table 16, for the appendicitis dataset, CVCF-SMOTE+FPSO-SVM achieves significantly better results than the best performance under NONE, SMOTE, SL-SMOTE, and B-SMOTE. However, it is not a significant difference for the best performance under SMOTE-TL.

From the experimental results, we see that CVCF-SMOTE+FPSO-SVM outperforms the compared algorithms for both the thoracic surgery dataset and the other two imbalanced datasets. On the one hand, it is because CVCF-improved SMOTE is well adapted to different datasets. On the other hand, FPSO-SVM automatically adjusts the optimal parameters according to different datasets, thus improving the generalization ability of the SVM.

### 3.5. Running Time Analysis

We compared the running time of CVCF-SMOTE+FPSO-SVM with the algorithms with the highest accuracy among all the compared methods. For the three datasets thoracic surgery, Haberman, and appendicitis, the algorithms with the highest accuracy among the compared methods are CVCF-SMOTE+GBDT, CVCF-SMOTE+KNN, and SMOTE-TL+FPSO-SVM, respectively. In addition, in order to compare the running time of FPSO-SVM with that of PSO-SVM, CVCF-SMOTE+PSO-SVM is also involved in the comparison. The comparison results are shown in Table 17. It can be seen from Table 17 that the running time for CVCF-SMOTE+FPSO-SVM is less than that of CVCF-SMOTE+PSO-SVM for the three datasets. However, the running time of CVCF-SMOTE+FPSO-SVM is slower than that of CVCF-SMOTE+GBDT, CVCF-SMOTE+KNN, and SMOTE-TL+FPSO-SVM for the thoracic surgery, Haberman, and appendicitis datasets, respectively. Considering the higher classification performance of our proposed method, it can still be considered superior to other algorithms.

The article "A Hybrid Method to Predict Postoperative Survival of Lung Cancer Using Improved SMOTE and Adaptive SVM" was published in 2021. Journal: Comput Math Methods Med.

## 4. Conclusion

In this work, we proposed a hybrid improved SMOTE and adaptive SVM method to predict the postoperative survival of LCPs. In our proposed hybrid model, CVCF is adopted to clear the data noise to improve the performance of SMOTE. Then, we use FPSO-optimized SVM to estimate whether the postoperative survival of LCPs is greater than one year. Experimental results show that our proposed CVCF-SMOTE+FPSO-SVM hybrid method obtains the best accuracy, *G*-mean, F1, and AUC as compared to other compared algorithms for postoperative survival prediction of LCPs.

Our proposed hybrid method can provide valuable medical decision-making support for LCPs and doctors. Considering the excellent classification performance for the other two imbalanced datasets, in the future, we will try to apply the proposed method to other problems based on imbalanced data, such as disease diagnosis and financial fraud detection. There are two limitations that need to be pointed out: one is that we only consider the 1-year survival after lung cancer surgery. In future studies, we will try to predict survival at other time points, such as survival 3 or 5 years after lung cancer surgery. The other is that the value range of the parameters of SVM in FPSO-SVM needs to be set manually, which may require some experience or experimental attempts. Designing a setting-free SVM is our future research direction.

## Figures and Tables

**Figure 1:** Using SMOTE alone may indiscriminately aggravate the noise.

**Figure 2:** Flowchart of the proposed hybrid method for predicting postoperative survival of LCPs.

**Figure 3:** Stacked histograms of accuracy, *G*-mean, F1, and AUC for different algorithms under different preprocessing methods.

**Figure 4:** ROC curve comparison of different algorithms under different preprocessing methods.

The article "A Hybrid Method to Predict Postoperative Survival of Lung Cancer Using Improved SMOTE and Adaptive SVM" was published in 2021. Journal: Comput Math Methods Med.

**Figure 5:** Fitness curves of FPSO-SVM (a) and PSO-SVM (b) with CVCF-SMOTE.

**Table 1:** Feature details of the thoracic surgery dataset.

Feature ID	Description	Type of attribute
1	Size of the original tumor, from OC11 (smallest) to OC14 (largest)	Nominal
2	Diagnosis (specific combination of ICD-10 codes for primary and secondary as well multiple tumors if any)	Nominal
3	Forced vital capacity	Numeric
4	Pain (presurgery)	Binary
5	Age at surgery	Numeric
6	Performance status	Nominal
7	Weakness (presurgery)	Binary
8	Dyspnoea (presurgery)	Binary
9	Cough (presurgery)	Binary
10	Haemoptysis (presurgery)	Binary
11	Peripheral arterial diseases	Binary
12	MI up to 6 months	Binary
13	Asthma	Binary
14	Volume that has been exhaled at the end of the first second of forced expiration	Numeric
15	Smoking	Binary
16	Type 2 diabetes mellitus	Binary
17	1-year survival period (true value if died)	Binary

**Table 2:** Confusion matrix.

	Actual positive	Actual negative
Predicted positive	TP	FP
Predicted negative	FN	TN

**Table 3:** Defuzzification of *w*, *c*_soc_, *c*_cog_, *η*, and *λ*.

Output	Level		
	Low	Medium	High
*w*	0.3	0.5	1.0
*c*_soc_	1.0	2.0	3.0
*c*_cog_	0.1	1.5	3.0
*λ*	0.0	0.001	0.01
*η*	0.1	0.15	0.2

**Table 4:** Accuracy comparison for different algorithms with different preprocessing methods.

Algorithms	NONE	SMOTE	SL-SMOTE	SMOTE-TL	B-SMOTE	CVCF-SMOTE
FPSO-SVM	**0.8440**	**0.7149**	**0.6385**	0.7378	**0.8679**	**0.9511**
PSO-SVM	**0.8440**	0.6570	0.6217	0.6776	0.7267	0.8643
SVM	**0.8440**	0.5294	0.5561	0.4781	0.5493	0.5204
RF	0.8369	**0.7149**	0.6023	**0.7388**	0.8430	0.8869
GBDT	0.8156	0.7059	0.5864	0.7025	0.8213	0.9276
KNN	0.8227	0.6561	0.5833	0.6910	0.7905	0.9005
AdaBoost	0.7943	0.6652	0.5615	0.6458	0.7674	0.9095

**Table 5:** *G*-mean comparison for different algorithms with different preprocessing methods.

Algorithms	NONE	SMOTE	SL-SMOTE	SMOTE-TL	B-SMOTE	CVCF-SMOTE
FPSO-SVM	0	0.6942	**0.6148**	0.7203	**0.8625**	**0.9510**
PSO-SVM	0	0.5832	0.5628	0.6150	0.6567	0.8501
SVM	0	0	0	0.1537	0.1015	0.1659
RF	0	**0.7092**	0.6017	**0.7385**	0.8404	0.8868
GBDT	**0.2938**	0.6901	0.5835	0.7024	0.8154	0.9274
KNN	0	0.6572	0.5819	0.6874	0.7919	0.9000
AdaBoost	0.2059	0.6550	0.5552	0.6464	0.7597	0.9096

**Table 6:** F1 comparison for different algorithms with different preprocessing methods.

Algorithms	NONE	SMOTE	SL-SMOTE	SMOTE-TL	B-SMOTE	CVCF-SMOTE
FPSO-SVM	0	0.6612	0.5549	0.7059	**0.8482**	**0.9502**
PSO-SVM	0	0.5089	0.4995	0.5600	0.6022	0.8336
SVM	0	0	0	0.2823	0.0605	0.0536
RF	0	**0.6834**	**0.5713**	**0.7458**	0.8241	0.8889
GBDT	**0.1333**	0.6524	0.5470	0.7025	0.7950	0.9292
KNN	0	0.6545	0.5473	0.7094	0.7760	0.9035
AdaBoost	0.0645	0.6186	0.5101	0.6425	0.7323	0.9099

The article "A Hybrid Method to Predict Postoperative Survival of Lung Cancer Using Improved SMOTE and Adaptive SVM" was published in 2021. Journal: Comput Math Methods Med.

**Table 7:** AUC comparison for different algorithms with different preprocessing methods.

Algorithms	NONE	SMOTE	SL-SMOTE	SMOTE-TL	B-SMOTE	CVCF-SMOTE
FPSO-SVM	0.5000	**0.7265**	**0.6268**	**0.7400**	**0.8639**	**0.9510**
PSO-SVM	0.5000	0.6426	0.6069	0.6754	0.7094	0.8631
SVM	0.5000	0.5000	0.5000	0.4993	0.5059	0.5138
RF	0.4958	0.7115	0.6038	0.7397	0.8411	0.8873
GBDT	**0.5202**	0.6993	0.5857	0.7052	0.8171	0.9281
KNN	0.4874	0.6581	0.5842	0.6919	0.7927	0.9010
AdaBoost	0.4891	0.6603	0.5582	0.6483	0.7621	0.9097

**Table 8:** Paired *t*-test results of CVCF-SMOTE+FPSO-SVM and the best performance under different preprocessing methods in terms of accuracy, F1, *G*-mean, and AUC on the thoracic surgery dataset. For CVCF-SMOTE, the *p* value is the statistic of the best result and the second best result.

Methods	Accuracy	F1	*G*-mean	AUC
NONE	11.034 (0.000)	25.502 (0.000)	21.102 (0.000)	27.01 (0.000)
SMOTE	14.348 (0.000)	16.01 (0.000)	10.261 (0.000)	12.469 (0.000)
SL-SMOTE	29.947 (0.000)	25.764 (0.000)	30.349 (0.000)	31.255 (0.000)
SMOTE-TL	29.815 (0.000)	30.281 (0.000)	22.248 (0.000)	26.895 (0.000)
B-SMOTE	6.541 (0.000)	5.176 (0.001)	5.297 (0.000)	5.997 (0.000)
CVCF-SMOTE	5.237 (0.001)	4.994 (0.001)	4.67 (0.001)	4.719 (0.001)

**Table 9:** Comparative results with previous studies based on accuracy.

Authors	Methods	Accuracy
Mangat and Vig [3]	DA-AC	82.18%
Elyan and Gaber [46]	RFGA	84.67%
Li et al. [47]	STDPNF	85.32%
Muthukumar and Krishnan [48]	IFSSs	88%
Saber Iraji [4]	ELM (wave kernel)	88.79%
Our work	CVCF-SMOTE+FPSO-SVM	95.11%

**Table 10:** Details of Haberman and appendicitis datasets.

Datasets	Case number	Attribute number	Class distribution
Haberman	306	3	225/81
Appendicitis	106	7	85/21

**Table 11:** Accuracy comparison for different algorithms with different preprocessing methods on the Haberman dataset.

Algorithms	NONE	SMOTE	SL-SMOTE	SMOTE-TL	B-SMOTE	CVCF-SMOTE
FPSO-SVM	**0.7402**	**0.6890**	0.6386	**0.7396**	**0.7795**	**0.8205**
PSO-SVM	0.7098	0.6435	**0.6504**	0.6538	0.6831	0.7205
SVM	0.7196	0.6291	0.6409	0.6423	0.6772	0.7165
RF	0.6989	0.6795	0.6142	0.7315	0.7559	0.7772
GBDT	0.6837	0.6606	0.6299	0.7252	0.7465	0.7764
KNN	0.7174	0.6630	0.6417	0.7000	0.7449	0.7992
AdaBoost	0.7163	0.6402	0.6331	0.6117	0.6819	0.7559

**Table 12:** AUC comparison for different algorithms with different preprocessing methods on the Haberman dataset.

Algorithms	NONE	SMOTE	SL-SMOTE	SMOTE-TL	B-SMOTE	CVCF-SMOTE
FPSO-SVM	0.5274	0.6813	0.6288	**0.7310**	**0.7748**	**0.8206**
PSO-SVM	0.5012	0.6131	0.6325	0.6669	0.6518	0.7121
SVM	0.5077	0.6096	0.6246	0.6598	0.6566	0.7035
RF	0.5731	**0.6815**	0.6132	0.7283	0.7588	0.7784
GBDT	0.5492	0.6607	0.6274	0.7226	0.7475	0.7765
KNN	0.5737	0.6649	**0.6418**	0.6997	0.7433	0.8009
AdaBoost	**0.5809**	0.6359	0.6293	0.6118	0.6779	0.7549

The article "A Hybrid Method to Predict Postoperative Survival of Lung Cancer Using Improved SMOTE and Adaptive SVM" was published in 2021. Journal: Comput Math Methods Med.

**Table 13:** Paired *t*-test results of CVCF-SMOTE+FPSO-SVM and the best performance under different preprocessing methods in terms of accuracy and AUC on the Haberman dataset.

Methods	Accuracy	AUC
NONE	6.603 (0.000)	18.744 (0.000)
SMOTE	6.555 (0.000)	10.315 (0.000)
SL-SMOTE	15.959 (0.000)	15.806 (0.000)
SMOTE-TL	4.506 (0.001)	3.539 (0.006)
B-SMOTE	2.601 (0.029)	2.83 (0.02)
CVCF-SMOTE	4.669 (0.001)	4.392 (0.002)

**Table 14:** Accuracy comparison for different algorithms with different preprocessing methods on the appendicitis dataset.

Algorithms	NONE	SMOTE	SL-SMOTE	SMOTE-TL	B-SMOTE	CVCF-SMOTE
FPSO-SVM	**0.8688**	**0.8792**	**0.8208**	**0.9381**	**0.9167**	**0.9511**
PSO-SVM	0.8625	0.8713	0.7620	0.8104	0.8714	0.9277
SVM	0.8469	0.7979	0.7854	0.8310	0.8813	0.9021
RF	0.8438	0.8438	0.7271	0.8714	0.9083	0.9106
GBDT	0.8188	0.8479	0.7146	0.8690	0.8917	0.9085
KNN	0.8500	0.7708	0.7354	0.8476	0.8708	0.8957
AdaBoost	0.8031	0.8396	0.7458	0.8690	0.8896	0.9106

**Table 15:** AUC comparison for different algorithms with different preprocessing methods on the appendicitis dataset.

Algorithms	NONE	SMOTE	SL-SMOTE	SMOTE-TL	B-SMOTE	CVCF-SMOTE
FPSO-SVM	0.6878	**0.8807**	**0.8167**	**0.9411**	**0.9135**	**0.9512**
PSO-SVM	0.5893	0.7602	0.7708	0.9311	0.8917	0.9239
SVM	0.6674	0.7966	0.7832	0.8423	0.8788	0.8982
RF	**0.6930**	0.8475	0.7324	0.8755	0.9064	0.9070
GBDT	0.6460	0.8539	0.7207	0.8713	0.8909	0.9092
KNN	0.6885	0.7736	0.7374	0.8499	0.8676	0.8954
AdaBoost	0.6352	0.8461	0.7492	0.8685	0.8888	0.9102

**Table 16:** Paired *t*-test results of CVCF-SMOTE+FPSO-SVM and the best performance under different preprocessing methods in terms of accuracy and AUC on the appendicitis dataset.

Methods	Accuracy	AUC
NONE	6.591 (0.000)	15.628 (0.000)
SMOTE	4.562 (0.001)	5.176 (0.001)
B-SMOTE	3.024 (0.014)	3.373 (0.008)
SL-SMOTE	6.227 (0.000)	7.009 (0.000)
SMOTE-TL	1.089 (0.304)	0.785 (0.453)
CVCF-SMOTE	2.764 (0.022)	2.787 (0.21)

**Table 17:** Running time (in second) by CVCF-SMOTE+FPSO-SVM and state-of-the-art algorithms.

Datasets	Algorithms		
Thoracic surgery	CVCF-SMOTE+GBDT	CVCF-SMOTE+PSO-SVM	CVCF-SMOTE+FPSO-SVM
	31.2	53.6	43.5

Haberman	CVCF-SMOTE+KNN	CVCF-SMOTE+PSO-SVM	CVCF-SMOTE+FPSO-SVM
	18.8	27.5	24.5

Appendicitis	SMOTE-TL+FPSO-SVM	CVCF-SMOTE+PSO-SVM	CVCF-SMOTE+FPSO-SVM
	13.8	22.2	17.3

## Data Availability

The dataset for this study can be obtained from the UCI machine learning database (http://archive.ics.uci.edu/ml/datasets/Thoracic+Surgery+Data).
